The article "Block Copolymer Nanomicelle-Encapsulated Curcumin Attenuates Cerebral Ischemia Injury and Affects Stem Cell Marker Expression by Inhibiting lncRNA GAS5" was retracted in 2024. Reasons: signs of a paper mill; suspected computer-generated content; unreliable results or conclusions; concerns about the data.

# Block Copolymer Nanomicelle-Encapsulated Curcumin Attenuates Cerebral Ischemia Injury and Affects Stem Cell Marker Expression by Inhibiting lncRNA GAS5

**DOI:** 10.1155/2023/9821500

**Published:** 2023-02-17

**Authors:** Fengguang Li, Yan Xu, Xinghua Wang, Xuan Cai, Wanli Li, Wei Cheng, Xing Li, Gangli Yan

**Affiliations:** ^1^Department of Neurology, Puren Hospital Affiliated to Wuhan University of Science and Technology, Wuhan, 430081 Hubei, China; ^2^Department of Pharmacy, General Hospital of Central Theater Command, Wuhan, 430010 Hubei, China

## Abstract

Stroke has become the most common cause of death among residents in China, among which ischemic stroke accounts for the vast majority reaching 70% to 80%. It is of great importance to actively investigate the protective mechanism of cerebral ischemia injury after IS (ischemic stroke). We constructed cerebral ischemia injury models *in vivo* MACO rat and *in vitro* (oxygen-glucose deprivation cell model) and set up different interference groups. RT-PCR (reverse transcription PCR) was conducted to detect the expression of lncRNA in neuronal cells, brain tissue, and plasma of different groups, and ELISA (enzyme-linked immunosorbent assay) and western blot were used to detect the expression of the protein in neuronal cells, brain tissue, and plasma of different groups. Cell activity was detected by the CCK-8 assay, while cell apoptosis was examined by TUNEL (terminal deoxynucleotidyl transferase dUTP nick end labeling) assay. In the rats' neuronal cells and brain tissue, curcumin can inhibit the expression of lncRNA GAS5 (long noncoding RNA growth arrest-specific 5). In oxygen-glucose-deprived neuronal cells *in vitro*, curcumin and low-expressed lncRNA GAS5 can enhance cell activity and decline cell apoptosis, but the addition of curcumin and overexpressed lncRNA GAS5 can make this phenomenon disappear. In neuronal cells, plasma, and brain tissue, curcumin and the low-expressed lncRNA GAS5 can inhibit the expression of IL-1*β* (interleukin 1 beta), TNF-*α* (tumor necrosis factor alpha), IL-6 (interleukin 6), Sox2 (SRY-box transcription factor 2), Nanog, and Oct4 (octamer-binding transcription factor 4). However, overexpressed lncRNA GAS5 and curcumin made the inhibitory effect disappear. In conclusion, this study demonstrated that curcumin could inhibit the expression of lncRNA GAS5, thereby inhibiting the expression of inflammation-related factors IL-1*β*, TNF-*α*, and IL-6, and ultimately achieve the purpose of attenuating cerebral ischemic cell damage. However, curcumin and lncRNA GAS5 may not alleviate cerebral ischemic cell damage by affecting stem cell differentiation.

## 1. Introduction

Stroke has become the most common cause of death in China [1] of which IS accounts for the vast majority, reaching 70% to 80% [2]. At present, the effective treatment methods for IS are mainly to open arteries and restore blood flow as soon as possible [3, 4] including intravenous thrombolysis and mechanical clot thrombectomy. However, due to the limitation of effective treatment time and other conditions, the vast majority of IS patients fail to receive these treatments. At the same time, the early vascular opening is not completely equivalent to a good curative effect, and the current statistical effective rate in the world is less than 50%. It is still of great importance to search for protective strategies for cerebral ischemia injury after IS.

The article "Block Copolymer Nanomicelle-Encapsulated Curcumin Attenuates Cerebral Ischemia Injury and Affects Stem Cell Marker Expression by Inhibiting lncRNA GAS5" was retracted in 2024. Reasons: signs of a paper mill; suspected computer-generated content; unreliable results or conclusions; concerns about the data.

Curcumin is a small molecule polyphenolic compound extracted from traditional Chinese medicine turmeric [5, 6]. It has anti-inflammatory, antioxidative stress, and antiapoptotic pharmacological effects [7]. It has an obvious protective effect on ischemic brain tissue [8]. However, due to its low water solubility, low uptake rate *in vivo*, and high blood clearance rate, curcumin has low bioavailability and cannot be used in clinical practice. Meanwhile, its neuroprotective mechanism of action has not been fully elucidated. Hydrophobic polycaprolactone (PCL) and hydrophilic polyethylene glycol (mPEG) copolymer carriers have low toxicity, high stability, and biodegradability. The natural polymer polyglutamic acid (PLG) can form an amphiphilic polymer with hydrophilic substances and can physically encapsulate hydrophobic drugs by using physical forces such as electrostatic adsorption or pi-pi stacking. Therefore, PLG-mPEG-PCL triblock polymer nanomicelles can be used as carrier materials to achieve the solubility and controlled release of curcumin.

Long noncoding RNAs (lncRNAs) are noncoding RNAs. The length of these noncoding RNA was found more than 200 nt. They have powerful regulatory roles including not only transcriptional regulation but also posttranscriptional regulation and chromatin modification [9]. In addition, lncRNAs can also regulate a variety of biological processes. Their abnormal expression may trigger various neurodegenerative diseases, such as parkinsonism [10], multiple sclerosis (MS) [11], and IS [12, 13]. It has been reported that lncRNAs, specifically growth arrest-specific transcript 5 (GAS5), affect neuronal apoptosis and function in IS [12]. Moreover, highly expressed GAS5 is not only associated with an increased risk of IS but also promotes neuronal apoptosis after cerebral infarction [14, 15]. GAS5 plays a critical role in various human cancers [16]. However, the effect of curcumin on lncRNA GAS5 is rarely reported. Therefore, the regulation of curcumin on lncRNA GAS5 is also included in this study. This research also explores whether curcumin can affect ischemic injury through lncRNA GAS5.

The article "Block Copolymer Nanomicelle-Encapsulated Curcumin Attenuates Cerebral Ischemia Injury and Affects Stem Cell Marker Expression by Inhibiting lncRNA GAS5" was retracted in 2024. Reasons: signs of a paper mill; suspected computer-generated content; unreliable results or conclusions; concerns about the data.

Despite advances in innovative treatment strategies, stroke remains one of the leading causes of death and disability worldwide. Due to significant therapeutic effects on patients with stroke, stem cell therapy has received extensive attention. Various types of cells (bone marrow mononuclear cells, bone marrow/adipose-derived stem/stromal cells, umbilical cord blood cells, neural stem cells, and olfactory ensheathing cells) have been shown to improve neurological function in animal models of stroke [17]. Therefore, in this study, we also tested some stem cell markers to explore the possible regulatory relationship among curcumin, lncRNA GAS5, and stem cell markers which have never been reported before. In this study, rats' neurons were first extracted and treated with glucose and oxygen deprivation. Multiple interference groups were set up, and we explored the regulatory relationship between curcumin and lncRNA GAS5 at the same time; their effects on inflammation-related factors, cell activity, and stem cell markers were also explored. This was further verified in animals. Curcumin and lncRNA GAS5 effects on cerebral ischemic cell damaging by affecting stem cell differentiation have been revealed in this study.

## 2. Materials and Methods

### 2.1. Preparation of Curcumin Nanomicelles Encapsulated by Triblock Copolymer

mPEG was grafted on the PLG segment through esterification reaction, a certain amount of *ε*-CL and mPEG was put into a dry polymerization tube treated with silicon chemical treatment, and we added catalyst Sn(Oct)2 and kept stirring it gently at 130°C for 6 hours. After vacuum degassing, cooling, purification, and drying, it was stored in a closed container for later use. Copolymer characterization tests were then performed. Hydrogen nuclear magnetic resonance (1H NMR) was first characterized by NMR (nuclear magnetic resonance) and relative molecular mass. The polymer thermal properties were then investigated with a NETZSCH DSC 204F1 instrument. The samples were then pressed with potassium bromide (KBr) and tested for infrared spectra on an FT-IR Spectrum BX infrared spectrometer. Dynamic light scattering (DLS) was performed by a Wyatt QELS instrument (Wyatt Technology) with a vertically polarized He-Ne laser (at 90°C) for detecting particle size and potential. Finally, fluorescence probe spectroscopy was used to detect the critical micelle concentration (CMC). Pyrene was used as a probe. Fluorescent probe technology was used to detect the ratio of CMC value. It was also used for the detection of the CMC value of mixed micelles of three groups (amphiphilic polymers with different hydrophilic block ratios).

The article "Block Copolymer Nanomicelle-Encapsulated Curcumin Attenuates Cerebral Ischemia Injury and Affects Stem Cell Marker Expression by Inhibiting lncRNA GAS5" was retracted in 2024. Reasons: signs of a paper mill; suspected computer-generated content; unreliable results or conclusions; concerns about the data.

An appropriate amount of curcumin and PLG-mPEG-PCL dissolved in acetone was used as a lipid phase, and an appropriate amount of poloxamer was dissolved in ultrapure water to form an aqueous phase. The lipid and aqueous phases were installed in separate tubes, and a syringe pump was set to inject the lipid and aqueous phases into the microchannels at a specific flow rate. The effluent was collected and centrifuged at low temperature and high speed for 30 min. The precipitate was ultrasonically dispersed in an appropriate amount of distilled water and then was freeze-dried for 24 h to obtain powdered curcumin nanoparticles which were stored at 4°C in the dark.

### 2.2. Identification of Triblock Copolymer-Encapsulated Curcumin Nanomicelles

Transmission electron microscopy (TEM) was used to observe the morphologies of blank micelles and drug-loaded micelles. Encapsulation efficiency (EE) and drug loading (LC) were determined. The drug release of the drug-loaded micelles was measured under physiological conditions, the concentration of curcumin was measured by UV light, and the cumulative drug release rate was calculated to obtain the in vitro release curve. A certain concentration of curcumin-loaded micelles was added to the VSMCs (vascular smooth muscle cells); cell culture medium and MTT (3-(4,5-dimethylthiazol-2-yl)-2,5-diphenyl-2H-tetrazolium bromide) analyses were performed to calculate the relative cell viability. Subsequently, *in vivo* pharmacokinetic assays were performed. The drug-containing rats' plasma samples, blank rats' plasma samples, and curcumin methanol control solution were taken, and the plasma curcumin content was analyzed by HPLC (high-performance liquid chromatography), and the relevant pharmacokinetic parameters were obtained by calculation. The same batch of polymer micelle solution/lyophilized powder formulation was left standing at different temperatures for a long time (4°C and normal temperature). Samples were taken at regular intervals to measure drug encapsulation efficiency, particle size, and particle size distribution. The above data changes were used to analyze its long-term stability.

### 2.3. Culture and Identify Primary Rat Hippocampal Neurons

SD (Sprague–Dawley) rats were purchased and bred. Rat hippocampal neurons were isolated from SD rats within 24 h of the newborn and placed in a 37°C CO_2_ incubator which was kept being cultured for 7 days with medium changes every three days. Neurons were identified *in vitro* using neuron-specific diluteolase (NSE) for subsequent experiments.

The article "Block Copolymer Nanomicelle-Encapsulated Curcumin Attenuates Cerebral Ischemia Injury and Affects Stem Cell Marker Expression by Inhibiting lncRNA GAS5" was retracted in 2024. Reasons: signs of a paper mill; suspected computer-generated content; unreliable results or conclusions; concerns about the data.

### 2.4. Oxygen-Glucose Deprivation (OGD) Model Establishment

The rat hippocampal neurons were placed in the MIC-101 (molecular incubator chamber-101) anaerobic culture system. The hypoxic chamber was connected to nitrogen, and the conditions were 95% N and 25% CO_2_. After being placed in a constant temperature incubator at 37°C for 3 hours, the sugar-free DMEM was replaced with a neuron medium (98% neurobasal medium+2% B27), and the rat hippocampal neurons were replaced in a CO_2_ incubator under normoxic concentration at 37°C, 5% for 6-24 h.

### 2.5. Construct lncRNA GAS5 Overexpression/Knockout Vector by CRISPR/Cas9 Technology

We designed the oligo DNA sequence of CRISPR/Cas9. sgRNA plasmid was constructed, transformed, and inoculated, and clones were picked. Plasmid DNA was extracted, and single-stranded oligonucleotides against the target gene locus were synthesized. The plasmid was electrotransfected into cells. 24 hours after transfection, the transfection efficiency was detected by qRT-PCR for subsequent experiments. The cells were divided into different groups: the control group (control), the model group (copolymer), the model+curcumin nanomicelle group (CC), the model+lncRNA GAS5 interference group (copolymer+GAS5 inhibitor), the model+lncRNA GAS5 overexpression group (copolymer+GAS5-plasmid), the model+curcumin nanomicelles+lncRNA GAS5 overexpression group (CC+GAS5-plasmid), and the model+curcumin nanomicelles+lncRNA GAS5 interference group (CC+GAS5 inhibitor). Among them, curcumin nanomicelles (concentration of 50 *μ*M) were added to the medium of the intervention group supplemented with curcumin nanomicelles.

### 2.6. The CCK8 Assay

The survival rate of cortical neurons was measured by the CCK8 method for 24 h after oxygen and glucose deprivation. Cells were seeded according to the instructions. Fresh medium (100 *μ*L) containing CCK8 solution (10 *μ*L) was added to each well of the 96-well plate in the dark and placed in an incubator to incubate in the dark for 2 h. After that, the cell proliferation rate was detected at 450 nm using a microplate reader.

### 2.7. TUNEL

Cell apoptosis was analyzed using a one-step TUNEL apoptosis detection kit (Beyotime, Shanghai, China) [18]. FITC's (fluorescein isothiocyanate) image is marked (green) in fluorescence microscopy. The green label indicates apoptotic cells. The nucleus was labeled blue with DAPI (Invitrogen™ D1306).

### 2.8. ELISA

The cytokine levels such as IL-1*β*, IL-6, and TNF-*α* in cells, plasma, and brain tissue of each group were detected by ELISA (Invitrogen™ Cat. No. CNB0011). The specific operation method was referred to in the kit instructions.

The article "Block Copolymer Nanomicelle-Encapsulated Curcumin Attenuates Cerebral Ischemia Injury and Affects Stem Cell Marker Expression by Inhibiting lncRNA GAS5" was retracted in 2024. Reasons: signs of a paper mill; suspected computer-generated content; unreliable results or conclusions; concerns about the data.

### 2.9. RT-PCR

The RNA from cells, plasma, and brain tissue was extracted by TRIzol kit procedure (Invitrogen™ TRIzol™ Reagent 15596026), and cDNA was synthesized by reverse transcription (Invitrogen™ M-MLV Reverse Transcriptase 28025013) after passing the quality inspection, and the PCR reaction system was configured to detect the mRNA expression of lncRNA GAS5. The primer sequences are lncRNA GAS5 forward-5′-TCT AGC TTG GGT GAG GCA-3′ and reverse-5′-TGG AGA GTC GGC TTG ACT A-3′;GAPDH forward-5′-ACG GAT TTG GTC GTA TTG G-3′ and reverse-5′-TCC CGT TCT CAG CCT TG-3 ′; lncRNA GAS5 forward-5′-TCT AGC TTG GGT GAG GCA-3′ and reverse-5′-TGG AGA GTC GGC TTG ACT A-3′; and GAPDH forward-5′-ACG GAT TTG GTC GTA TTG G-3′ and reverse-5′-TCC CGT TCT CAG CCT TG-3′. For 50 *μ*L total volume, the following PCR recipe was used: 10x buffer 4 *μ*L, 50 mM MgCl_2_ 2.5 *μ*L, amplification primer 1 (10 *μ*M) 0.9 *μ*L, amplification primer 2 (10 *μ*M) 0.9 *μ*L, Taq DNA polymerase (5 U/*μ*L) 0.5 *μ*L, cDNA 2.2 *μ*L, and dis.H_2_O 39 *μ*L. For the PCR profile, initial denaturation was done at 94°C, denaturation at 96°C, annealing at 56°C, elongation at 71°C, and final elongation at 72°C.

### 2.10. Western Blot

The proteins in cells and tissues were extracted. The concentration of protein was determined by BCA (bicinchoninic acid) method. We prepared 10% SDS-PAGE, loaded an equal amount of protein sample, and performed electrophoresis at 90 V. The protein on the gel was transferred to a PVDF (polyvinylidene fluoride) membrane. This membrane was removed and blocked in a 10% nonfat milk-blocking solution. TBST (Tris-buffered saline with Tween 20) was used for membrane washing. After washing, it was incubated with primary antibody (Sox2, 1 : 1500, ab92494, Abcam; Nanog, 1 : 1500, ab109250, Abcam; and Oct4, 1 : 1000, ab181557, Abcam) overnight at 4°C. The membrane was washed with TBST and incubated with a secondary antibody (goat anti-rabbit IgG H&L (HRP), 1 : 5000, ab6721, Abcam) for 2 h at room temperature. The membrane was washed with TBST. The PVDF membrane was placed in a dark room. ECL color developing working solution was added dropwise for development. The protein expression of Sox2, Nanog, and Oct4 was detected [18].

### 2.11. Animal Experiment

A total of 72 8-week-old SPF-grade healthy male SD rats with a weight between 250 and 280 g were selected and divided into groups: sham operation group (sham), model group (copolymer), model+curcumin nanomicelle group (CC), model+lncRNA GAS5 interference group (copolymer+GAS5 inhibitor), model+lncRNA GAS5 overexpression group (copolymer+GAS5-plasmid), model+curcumin nanomicelles+lncRNA GAS5 overexpression group (CC+GAS5-plasmid), and model+curcumin nanomicelles+lncRNA GAS5 interference group (CC+GAS5 inhibitor). The model+curcumin nanomicelle group was 80 mg/kg (body weight), with 12 mice in each group. The control group and the model group were fed with water normally before the operation.

The article "Block Copolymer Nanomicelle-Encapsulated Curcumin Attenuates Cerebral Ischemia Injury and Affects Stem Cell Marker Expression by Inhibiting lncRNA GAS5" was retracted in 2024. Reasons: signs of a paper mill; suspected computer-generated content; unreliable results or conclusions; concerns about the data.

### 2.12. Preparation of Ischemic Stroke (Suture Method MACO) Model

The model groups were fed the corresponding drugs by gavage for 14 days before modeling. To analyze the impairment of neurons in SD rats, MACO model was established [19]. Two groups named as operation and sham were used in the model. In the operation group, the right middle cerebral artery was blocked by a suture to achieve focal cerebral ischemia, and the wound was sutured. Rats were kept in a single cage after the operation, and the suture was gently withdrawn from the ICA 2 hours later to realize reperfusion. In the sham-operated group, only the right carotid artery was isolated, no suture was inserted, and no neurological damage was observed after the operation.

The success criteria of the model were wrist-elbow flexion and shoulder internal rotation of the right forelimb and inability to stretch forward grasp or tilt to the opposite side. Rats with no neurological impairment and subarachnoid hemorrhage were excluded.

Neurobehavioral scores were used to judge the animal models. The Zea-longa scoring method was used. 0-4 score was given according to the level of neural damage. Scores between 1 and 3 indicated successful modeling, and rats with scores of 0 and 4 were excluded. The 0 score indicated the no impairment in neural functions, while 4 score represented the acute damage in the neural functions.

### 2.13. Statistical Methods

The experimental data of this study were statistically analyzed by using GraphPad software (https://www.graphstats.net/graphpad-prism). Differences between the two groups (control and experimental or model) were calculated using an unpaired *t*-test. When *P* value < 0.05, this means the difference is statistically significant.

## 3. Results

To investigate the protective mechanism of cerebral ischemia injury after IS. Cerebral ischemia injury models *in vivo* MACO rat and *in vitro* (oxygen-glucose deprivation cell model) were constructed. The expressions of lncRNA in neuronal cells, brain tissue, and plasma were detected by RT-PCR. The expression of the protein in neuronal cells, brain tissue, and plasma was determined by ELISA and western blot. Cell activity was detected by the CCK-8 assay. TUNEL assay determines cell apoptosis. Curcumin can inhibit the expression of lncRNA GAS5 in the rats' neuronal cells and brain tissue. In neuronal cells, plasma, and brain tissue, curcumin and the low-expressed lncRNA GAS5 can inhibit the expression of IL-1*β*, TNF-*α*, IL-6, Sox2, Nanog, and Oct4.

The article "Block Copolymer Nanomicelle-Encapsulated Curcumin Attenuates Cerebral Ischemia Injury and Affects Stem Cell Marker Expression by Inhibiting lncRNA GAS5" was retracted in 2024. Reasons: signs of a paper mill; suspected computer-generated content; unreliable results or conclusions; concerns about the data.

The spherical-shaped nanomicelles were observed by TEM. The mean diameter of the nanomicelles was less than 53 nm, while calculated value for zeta potential was +42.1. Change in the size of nanomicelles evaluated the encapsulation of curcumin nanomicelle while the encapsulation process was confirmed by various assays, which showed the decreased expression of lncRNA GAS5.

### 3.1. Triblock Copolymer-Encapsulated Curcumin Nanomicelles Inhibit lncRNA GAS5 Expression

To verify the effects of lncRNA GAS5 inhibitor and lncRNA GAS5 plasmids on lncRNA GAS5 expression, we first verified their transfection efficiency in cells. The results demonstrated that the lncRNA GAS5 inhibitor could significantly inhibit the expression of lncRNA GAS5 (Figure 1(a)), while the lncRNA GAS5 plasmid could significantly upregulate the expression of lncRNA GAS5 (Figure 1(b)). Subsequently, we set up different interference groups to explore the effect of triblock copolymer-encapsulated curcumin nanomicelles on the expression of lncRNA GAS5. The results showed that curcumin nanomicelles encapsulated by triblock copolymers could significantly inhibit the expression of lncRNA GAS5 (Figure 1(c)).

### 3.2. Triblock Copolymer-Encapsulated Curcumin Nanomicelles Enhance Cell Viability and Inhibit the Expression of IL-1*β*, TNF-*α*, and IL-6 via lncRNA GAS5

To explore the effect of triblock copolymer-encapsulated curcumin on cell viability, we conducted cell viability experiments. The results showed that both triblock copolymer-encapsulated curcumin nanomicelles and low-expressed lncRNA GAS5 could enhance cell viability. But in the triblock copolymer-encapsulated curcumin nanomicelles and the lncRNA GAS5 interference group (CC+GAS5-plasmid), the enhancement effect disappeared (Figure 2(a)). It can be inferred that the curcumin nanomicelles encapsulated by triblock copolymers enhance cell activity by inhibiting the expression of lncRNA GAS5. Subsequently, to explore the effect of triblock copolymer-encapsulated curcumin on ischemic injury, we interfered with the cells after hypoxia deprivation and detected the expressions of IL-1*β*, TNF-*α*, and IL-6 by the ELISA experiment. The results showed that triblock copolymer-encapsulated curcumin nanomicelles and low-expressed lncRNA GAS5 significantly inhibited the expression of IL-1*β* (Figure 2(b)), TNF-*α* (Figure 2(c)), and IL-6 (Figure 2(d)). However, in the triblock copolymer-encapsulated curcumin nanomicelles and lncRNA GAS5 interference group (CC+GAS5-plasmid), this inhibitory effect disappeared. This proved that the block copolymer-encapsulated curcumin nanomicelles inhibited the expression of IL-1*β*, TNF-*α*, and IL-6 by inhibiting the lncRNA GAS5. The result of the TUNEL assay showed that both triblock copolymer-encapsulated curcumin nanomicelles and low-expressed lncRNA GAS5 could decrease cell apoptosis. But in the triblock copolymer-encapsulated curcumin nanomicelles and the lncRNA GAS5 interference group (CC+GAS5-plasmid), the effect disappeared (Figure 2(e)).

The article "Block Copolymer Nanomicelle-Encapsulated Curcumin Attenuates Cerebral Ischemia Injury and Affects Stem Cell Marker Expression by Inhibiting lncRNA GAS5" was retracted in 2024. Reasons: signs of a paper mill; suspected computer-generated content; unreliable results or conclusions; concerns about the data.

### 3.3. Triblock Copolymer-Encapsulated Curcumin Nanomicelles Inhibit the Expression of Stem Cell Markers by Inhibiting lncRNA GAS5

To explore the effect of triblock copolymer-encapsulated curcumin nanomicelles and lncRNA GAS5 on stem cells, we detected stem cell markers. The results showed that curcumin nanomicelles encapsulated by triblock copolymers can inhibit the expression of stem cell markers Sox2 (Figure 3(a)), Nanog (Figure 3(b)), and Oct4 (Figure 3(c)) and inhibit the expression of lncRNA GAS5 achieving the same effect. According to the previous results, triblock copolymer-encapsulated curcumin nanomicelles can downregulate the expression of lncRNA GAS5. Therefore, we speculate that curcumin nanomicelles encapsulated by triblock copolymers can regulate stem cell markers by inhibiting lncRNA GAS5. The expression of Sox2 (Figure 3(a)), Nanog (Figure 3(b)), and Oct4 (Figure 3(c)) in the CC+GAS5-plasmid group and the control group was not significantly different, which also confirmed this.

### 3.4. The Effect of Triblock Copolymer-Encapsulated Curcumin Nanomicelles on lncRNA GAS5 in Animals and Its Subsequent Influence

To verify whether the regulation of lncRNA GAS5 by triblock copolymer-encapsulated curcumin nanomicelles and its subsequent effects in animals were consistent with the previous cell experiments, we conducted follow-up animal experiments. Animal models were judged using behavioral scores, and mice with scores 1-4 were selected for follow-up studies (Figure 4(a)). The transfection effect in animals of the interference group was verified, the expression of lncRNA GAS5 in different interference groups was detected, and the results were consistent with expectations (Figure 4(b)).

Plasma and brain tissue were extracted for detection. Plasma results showed that curcumin nanomicelles encapsulated by triblock copolymer and low-expressed lncRNA GAS5 could significantly inhibit the expression of cytokines IL-1*β*, TNF-*α*, and IL-6 (Figures 5(a)–5(c)).

After upregulating the expression of lncRNA GAS5, this inhibitory effect was also alleviated. Similar results were obtained after testing brain tissue. In brain tissue, curcumin nanomicelles encapsulated by triblock copolymer and low-expressed lncRNA GAS5 can also significantly inhibit the expression of cytokines IL-1*β*, TNF-*α*, and IL-6 (Figures 5(d)–5(f)), while this inhibitory effect was also alleviated after upregulating the expression of lncRNA GAS5.

The article "Block Copolymer Nanomicelle-Encapsulated Curcumin Attenuates Cerebral Ischemia Injury and Affects Stem Cell Marker Expression by Inhibiting lncRNA GAS5" was retracted in 2024. Reasons: signs of a paper mill; suspected computer-generated content; unreliable results or conclusions; concerns about the data.

Subsequently, we detected stem cell markers in plasma and brain tissue. Plasma results showed that curcumin nanomicelles encapsulated by triblock copolymers could inhibit the expression of stem cell markers Sox2, Nanog, and Oct4 (Figures 6(a)–6(c)). The low-expressed lncRNA GAS5 can inhibit the expression of Sox2, Nanog, and Oct4, while the high-expressed lncRNA GAS5 can promote the expression of Sox2, Nanog, and Oct4 (Figures 6(a)–6(c)). The expression of curcumin nanomicelles encapsulated by triblock copolymers and overexpressed lncRNA GAS5, Sox2, Nanog, and Oct4 had no significant difference from the control group. Brain tissue results also showed that curcumin nanomicelles encapsulated by triblock copolymers could inhibit the expression of stem cell markers Sox2, Nanog, and Oct4 (Figures 6(d)–6(f)). Similar results can be achieved by inhibiting the expression of lncRNA GAS5. Similarly, curcumin nanomicelles encapsulated by triblock copolymers and overexpressed lncRNAs GAS5, Sox2, Nanog, and Oct4 showed no significant difference from the control group (Figures 6(d)–6(f)). The above results were consistent with the results of cell experiments, indicating that curcumin nanomicelles encapsulated by triblock copolymers can regulate the expression of lncRNA GAS5, and affect the expression of cytokines and stem cell markers by regulating lncRNA GAS5.

## 4. Discussion

Through experiments in rats' neuronal cells, we found that curcumin can inhibit the expression of lncRNA GAS5. In addition, curcumin can also increase the cell activity of neuronal cells after the glucose-oxygen deprivation experiment, and inhibiting the expression of lncRNA GAS5 can also achieve the result of enhancing cell activity. This was similar to previous reports that curcumin and lncRNA GAS5 can promote cell survival [20–22]. Expression levels of GAS5 in various tumors have been studied [16]. However, adding curcumin while overexpressing the lncRNA GAS5 made this effect disappear. This indicated that curcumin enhances cell activity by inhibiting lncRNA GAS5.

Ischemic stroke can be caused by a variety of factors, such as cardiogenic embolism, occlusion of small cerebral vessels, and atherosclerosis affecting cerebral circulation. There is increasing evidence that the immune system plays a complex role in the pathophysiological changes that occur after cerebral ischemic injury. Following ischemic brain injury, we can observe the ensuing neuroinflammation causing additional damage and triggering cell death [23–26]. Therefore, to further study the pathway by which curcumin and lncRNA GAS5 alleviated ischemic injury, we tested inflammation-related factors. We detected IL-1*β*, TNF-*α*, and IL-6 in rats' neuronal cells and rats' brain and plasma tissues. The results showed that both curcumin and low-expressed lncRNA GAS5 could inhibit the expression of IL-1*β*, TNF-*α*, and IL-6, and when lncRNA GAS5 was overexpressed, the inhibitory effect of curcumin on the expression of IL-1*β*, TNF-*α*, and IL-6 disappeared. This indicated that curcumin inhibited the expression of IL-1*β*, TNF-*α*, and IL-6 by inhibiting the expression of lncRNA GAS5. Previous studies have also reported that curcumin inhibits inflammatory factors IL-1*β*, TNF-*α*, and IL-6 [27–29], but we have found an intermediate regulatory lncRNA, which further explained curcumin's regulation of inflammatory factors. Finally, we tested some stem cell markers, Sox2, Nanog, and Oct4. The results showed that both curcumin and the low-expressed lncRNA GAS5 could inhibit the expression of Sox2, Nanog, and Oct4, which was similar to previous reports [19, 22, 29–32]. This suggests that perhaps curcumin cannot promote stem cell differentiation but only enhance cell survival [20]. The therapeutic effect of stem cells on ischemic stroke may not be regulated by curcumin.

The article "Block Copolymer Nanomicelle-Encapsulated Curcumin Attenuates Cerebral Ischemia Injury and Affects Stem Cell Marker Expression by Inhibiting lncRNA GAS5" was retracted in 2024. Reasons: signs of a paper mill; suspected computer-generated content; unreliable results or conclusions; concerns about the data.

## 5. Conclusion

In summary, this study established in vivo (rat MACO model) and in vitro (oxygen-glucose deprivation cell model) cerebral ischemia injury models and found that curcumin can inhibit the expression of lncRNA GAS5 in neuronal cells, plasma, and brain tissue. In addition, curcumin inhibits the expression of inflammatory-related factors IL-1*β*, TNF-*α*, and IL-6 by inhibiting its expression and finally achieves the purpose of alleviating cerebral ischemic cell damage. Curcumin and the low-expressed lncRNA GAS5 can enhance cell viability and decline cell apoptosis. In addition, curcumin and the low-expressed lncRNA GAS5 can also inhibit the expression of stem cell markers Sox2, Nanog, and Oct4. This indicates that curcumin and lncRNA GAS5 may not alleviate cerebral ischemic cell damage by affecting stem cell differentiation.

## Figures and Tables

**Figure 1:** Triblock copolymer-encapsulated curcumin nanomicelles downregulate lncRNA GAS5 expression. (a, b) Transfection efficiency detection. (c) Detection of the expression of lncRNA GAS5 through RT-PCR (^∗^*P* < 0.05, ^∗∗^*P* < 0.01, ^∗∗∗^*P* < 0.001, and ^∗∗∗∗^*P* < 0.0001; ns: not significant).

**Figure 2:** Cell viability and cytokine expression detections. (a) CCK-8 assay to detect cell activity. (b–d) The expression of cytokines IL-1*β* (b), TNF-*α* (c), and IL-6 (d) at the cellular level. (e) TUNEL assay to detect cell apoptosis (^∗^*P* < 0.05, ^∗∗^*P* < 0.01, and ^∗∗∗^*P* < 0.001; ns: not significant).

The article "Block Copolymer Nanomicelle-Encapsulated Curcumin Attenuates Cerebral Ischemia Injury and Affects Stem Cell Marker Expression by Inhibiting lncRNA GAS5" was retracted in 2024. Reasons: signs of a paper mill; suspected computer-generated content; unreliable results or conclusions; concerns about the data.

**Figure 3:** Low-expressed lncRNA GAS5 promotes the expression of stem cell markers. (a–c) The expression of stem cell markers Sox2 (a), Nanog (b), and Oct4 (c) at the cellular level (^∗^*P* < 0.05, ^∗∗^*P* < 0.01, and ^∗∗∗^*P* < 0.001; ns: not significant).

**Figure 4:** Animal modeling evaluation and lncRNA GAS5 detection. (a) Animal model scoring. (b) Detection of the expression of lncRNA GAS5 through RT-PCR (^∗^*P* < 0.05, ^∗∗^*P* < 0.01, ^∗∗∗^*P* < 0.001, and ^∗∗∗∗^*P* < 0.0001; ns: not significant).

**Figure 5:** Triblock copolymer-encapsulated curcumin nanomicelles regulate the expression of GAS5-induced cytokines. (a–c) The expression of cytokines IL-1*β* (a), TNF-*α* (b), and IL-6 (c) in plasma. (d–f) The expression of cytokines IL-1*β* (d), TNF-*α* (e), and IL-6 (f) in brain tissue (^∗^*P* < 0.05, ^∗∗^*P* < 0.01, and ^∗∗∗^*P* < 0.001; ns: not significant).

**Figure 6:** Triblock copolymer-encapsulated curcumin nanomicelles inhibit the expression of stem cell markers. (a–c) The expression of stem cell markers Sox2 (a), Nanog (b), and Oct4 (c) in plasma. (d–f) The expression of stem cell markers Sox2 (d), Nanog (e), and Oct4 (f) in brain tissue (^∗^*P* < 0.05, ^∗∗^*P* < 0.01, and ^∗∗∗^*P* < 0.001; ns: not significant).

## Data Availability

The data used to support the findings of this study are included within the article.
